The article "Research on Teaching Resource Recommendation Algorithm Based on Deep Learning and Cognitive Diagnosis" was published in 2022. Journal: J Healthc Eng.

# Research on Teaching Resource Recommendation Algorithm Based on Deep Learning and Cognitive Diagnosis

**DOI:** 10.1155/2022/5776341

**Published:** 2022-01-07

**Authors:** Fei Zhou

**Affiliations:** School of Computer, Huanggang Normal University, Hubei, Huanggang 438000, China

## Abstract

With the increasing abundance of network teaching resources, the recommendation technology based on network is becoming more and more mature. There are differences in the effect of recommendation, which leads to great differences in the effect of recommendation algorithms for teaching resources. The existing teaching resource recommendation algorithm either takes insufficient consideration of the students' personality characteristics, cannot well distinguish the students' users through the students' personality, and pushes the same teaching resources or considers the student user personality not sufficient and cannot well meet the individualized learning needs of students. Therefore, in view of the above problem, combining TDINA model by the user for the students to build cognitive diagnosis model, we put forward a model based on convolution (CUPMF) joint probability matrix decomposition method of teaching resources to recommend the method combined with the history of the students answer, cognitive ability, knowledge to master the situation, and forgetting effect factors. At the same time, CNN is used to deeply excavate the test question resources in the teaching resources, and the nonlinear transformation of the test question resources output by CNN is carried out to integrate them into the joint probability matrix decomposition model to predict students' performance on the resources. Finally, the students' knowledge mastery matrix obtained by TDINA model is combined to recommend corresponding teaching resources to students, so as to improve learning efficiency and help students improve their performance.

## 1. Quotation

In recent years, with the development of online education and intelligent teaching, the era of big data in education Internet plus has been ushered in, and both the number of users and the number of teaching resources have exploded. In the actual teaching system, students cannot spend a lot of time learning massive teaching resources, and it is unnecessary. The most important thing is to choose teaching resources that are more in line with students' individual needs by understanding students' cognitive ability and learning situation, so as to help students review, consolidate, and improve their knowledge. In today's personalized online education platform, teaching resource recommendation has gradually attracted the attention of more and more educational research scholars. How to recommend teaching resources for different students and users from massive teaching resources in a limited time has become a key problem [1] to be solved urgently.

The article "Research on Teaching Resource Recommendation Algorithm Based on Deep Learning and Cognitive Diagnosis" was published in 2022. Journal: J Healthc Eng.

The assessment of students' proficiency is very important in educational assessment, and the cognitive diagnostic model (CDM s) as we know it is a psychological tool for assessment. We propose a generalized multistrategy clean development mechanism for dichotomous response data. The model provides a framework that can adapt to various rule methods and adopts an expectation maximization algorithm [2]. Experiments show that the model is feasible and can recover the data well. Students' mastery of more skills plays an important role in employment development. More and more students want to learn a specific skill, which requires more courses and teaching tool libraries. Students spend a lot of time searching for these tools. Then it is very important for educators to help students choose in this respect. On the basis of previous transfer analysis and learning trajectory, we propose a new model, which makes students' acquisition of skills more dependent on the effectiveness of learning tools and their interaction with other skills, that is, a multilevel logistic hidden Markov learning model based on cognitive diagnosis model [3]. Culture and tourism industries are becoming more and more mature, so we need to study their integration. Neural network is widely used in the field of cognitive diagnosis. For cognitive diagnosis subjects, they can judge their status according to their reactions and their cognitive attributes and then put forward remedial schemes. At present, we regard cultural industry and tourism industry as independent individuals, establish a complementary system based on neural network algorithm, start from the perspective of blockchain, and make integrated diagnosis with rural culture and rural tourism industry, aiming at making certain contributions to the development of rural tourism [4].

Through experiments, we evaluate the influence of school teaching resources, including how to use them on students' grades. The change caused by the adjustment of funding is to reduce the funding for teaching resources and increase the funding for another school, which reflects that the schools with increased funding have improved students' grades without behavioral costs [5]. It also shows that increasing school week's increases homework time without reducing social and school satisfaction or increasing school violence. Based on the existing multiphase CDM, a cognitive diagnosis model CDMs with multidimensional scoring items is proposed. The feasibility and performance of the model in the simulation study surface, under different conditions, CDMs parameters can be better recovered. In addition, compared with CAIC and BIC, BIC has better performance in selecting the most suitable model. By analyzing the data, the application of CDMS is proved [6]. The learning management system of online teacher community is an online resource developed, which supports teachers in different fields to learn the advantages of their resources and contain realistic case experiences. The investigation shows the effectiveness of this resource [7]. The relevant literature is described above, but there are different degrees of influence on the recommendation effect of teaching resources. Teaching resource recommendation has a high cost, so it is necessary to compare the recommendation effect of different methods. The above methods are not given. Therefore, the recommendation method proposed in this paper has obvious advantages in recommendation effect.

The article "Research on Teaching Resource Recommendation Algorithm Based on Deep Learning and Cognitive Diagnosis" was published in 2022. Journal: J Healthc Eng.

## 2. Algorithm Design of TDINA Model

At present, in most classroom teaching or online education platforms and smart classrooms, students and users are usually tested through traditional examination papers [8]. The test results only reflect students' scores, but cannot reflect students' cognitive process, knowledge structure, and cognitive ability level through specific answer situations, and lack of in-depth mining mechanism for students' answer situations. By constructing an accurate algorithm model to obtain students' user knowledge and ability level, we can improve the understanding of students' cognitive ability level at present, and it is also the key to solve such problems. The cognitive diagnosis theory developed by combining educational psychometrics with cognitive psychology provides a powerful solution to this problem. Cognitive diagnosis theory is generally included on the basis of cognitive attribute *Q* matrix. Cognitive diagnosis model can further identify the potential knowledge state and cognitive ability level of the tested (generally referring to student users), such as the proficiency of specific skills, and finally evaluate the knowledge ability level of the tested, so as to describe and model them. The most widely used cognitive diagnosis models mainly include item response theory (IRT) model and potential classification model (DINA model) [9]. Among them, DINA model describes student users as a multidimensional knowledge point mastery vector and diagnoses them according to students' actual answers. DINA model can solve the problem that a single test item involves multiple attribute skills, and its parameters can be interpreted well. At the same time, the complexity of the model is not affected by the number of attributes. However, the potential influencing factors considered in DINA model are not comprehensive. Therefore, according to the cognitive diagnosis technology of educational psychology, combined with students' historical answer records, this study introduces influencing factors such as forgetting effect and answer times of knowledge-related resources, improves DINA model in the calculation of key positive answer rate, and proposes a time-sensitive deterministic input and noise gate (TDINA) model [10].

The article "Research on Teaching Resource Recommendation Algorithm Based on Deep Learning and Cognitive Diagnosis" was published in 2022. Journal: J Healthc Eng.

### 2.1. 1DINA Modeling

TDINA model belongs to the potential classification model of cognitive diagnosis model, which is suitable for cognitive diagnosis of binary scoring item test. The algorithm flow of TDINA model is shown in Figure 1, which can be divided into the following eight steps.

**Step 1 .**

Assume that the target student user is *u*_*i*_. According to the basic information of student user *u*_*i*_ (such as grade information and subject information), redundant data with small relationship are filtered to obtain an initial student user set *US* *=* *{u*_1_*, u*_2_*, u*_3_*,..., u*_*m*_*}*, a test set *TS* *=* *{t*_1_*, t*_2_*, t*_3_*,..., t*_*n*_*},* and a knowledge point set *KS* *=* *{k*_1_*, k*_2_*, k*_3_*,..., k*_*l*_*}*.

**Step 2 .**

In the behavior data (mainly answer data) collected by the system, the student-test score matrix is constructed and recorded as *R*_*m×n*_. The examination questions-knowledge points investigation matrix is constructed by some field subject experts in colleges and universities, which is recorded as *Q*_*n×m*_. Matrix *R* and Matrix *Q* are shown in Figure 2.

**Step 3 .**

Define that each student user *u*_*i*_ can obtain a knowledge point mastery vector area *α* *=* *{α*_*i1*_*, α*_*i2*_*, α*_*i3*_*… α*_*il*_*}*, where *α*_*ij*_ *=* *1* means that the student *u*_*i*_ grasps the knowledge point *k*_*j*_; *α*_*ij*_ *=* *0* means that the student *u*_*i*_ has not mastered the knowledge point *k*_*j*_. The ultimate goal of TDNA model is to find the mastery matrix *A* *=* {*α*_1_*, α*_2_*, α*_3_*… α*_*m*_} of students-knowledge points.

**Step 4 .**

Define the student's initial response as in (1), where *ε*_*ij*_  = 1 denotes the student user *u*_*i*_. Mastering the test *t*_*j*_, all the knowledge points are investigated. On the contrary, *ε*_*ij*_  = 0 means that the student user *u*_*i*_ has not fully mastered all the knowledge points examined in the test *t*_*j*_.

(1) $$\begin{array}{c} \begin{array}{c} \varepsilon_{\text{ij}}=\prod_{k=1}^{l}\alpha_{\text{ik}}^{q_{j}k} \end{array}. \end{array}$$

**Step 5 .**

Combined with the actual situation of student users, that is, when students answer a certain test question, there are some mistakes and guesses. Therefore, the error rate and guess rate are defined as Formulas 2 and (3), respectively.

(2) $$\begin{array}{c} \begin{array}{c} s_{j}=p\left(r_{\text{ij}}=0|\varepsilon_{\text{ij}}=1\right) \end{array}. \end{array}$$

(3) $$\begin{array}{c} \begin{array}{c} g_{j}=p\left(r_{\text{ij}}=1|\varepsilon_{\text{ij}}=0\right) \end{array}. \end{array}$$

**Step 6 .**

The article "Research on Teaching Resource Recommendation Algorithm Based on Deep Learning and Cognitive Diagnosis" was published in 2022. Journal: J Healthc Eng.

Combined with the formula and matrix defined in the previous step, calculate the positive answer rate *p(r*_*ij*_ *=* *1*｜*a*_*i*_) on the test *t*_*i*_ and express it with a formula such as

(4) $$\begin{array}{c} \begin{array}{c} p\left(r_{\text{ij}}=1|a_{i}\right)={\left(1-s_{j}\right)}^{\varepsilon_{\text{ij}}}g^{1-\varepsilon_{\text{ij}}} \end{array}. \end{array}$$

**Step 7 .**

From the perspective of students, students' positive answer rate to test questions changes with the constant changes of their own personalities. Students' own personality information has great influence on the calculation of correct answer rate. Among all students' personality information, some information is relatively stable, such as name, gender, and subject, but some information is constantly changing, such as the time of answering records, the number of answering knowledge points, and the mastery rate of knowledge points. The TDINA model proposed in this study takes into account the forgetting effect of students' answers to history questions and the memory consolidation effect of the times of answering questions *t*_*j*_, which are both functions of time. Based on this, this paper introduces these two factors into the time factor *τ*_*j*_, to improve the DINA model, in which the definition of time factor is as

(5) $$\begin{array}{c} \begin{array}{c} \tau_{j}=T\left(\lambda ,\alpha ,\beta \right)=\frac{\sum \beta \left(1-\lambda t^{\alpha }\right)}{\text{count}\left(\beta \right)} \end{array}, \end{array}$$

where *λ* and *α* are constant parameters, which are used to fit Ebbinghaus forgetting curve, and *β* parameter is the situation that students answer questions *t*_*j*_ in history; if students answer correctly, it is 1; otherwise, the value is 0. count (B) indicates the number of times students answer questions *t*_*i*_, and the final formula of students' positive answer rate is (6) combined with the positive answer rate in Step 6.

(6) $$\begin{array}{c} p\left(t_{\text{ij}}=1|a_{i}\right)=T\left(\lambda ,\alpha ,\beta \right){\left(1-s_{i}\right)}^{\varepsilon_{\text{ij}}}g_{j}^{1-\varepsilon_{\text{ij}}}=\frac{\sum \beta \left(1-\lambda t^{\alpha }\right)}{\text{count}\left(\beta \right)}{\left(1-s_{j}\right)}^{\varepsilon_{\text{ij}}}g_{j}^{1-\varepsilon_{\text{ij}}}. \end{array}$$

**Step 8 .**

The article "Research on Teaching Resource Recommendation Algorithm Based on Deep Learning and Cognitive Diagnosis" was published in 2022. Journal: J Healthc Eng.

The edge likelihood in (6) is maximized by EM algorithm, and the maximum likelihood estimator of sky carbon rate and the maximum likelihood estimator of guess rate are obtained. Finally, the maximum a posteriori probability algorithm is used to obtain the knowledge point mastery vector estimator of the student user.

## 3. Design of Recommendation Algorithm for CUPMF Model

### 3.1. Overall Framework

The teaching resource recommendation method based on convolution joint probability matrix factorization (CUPMF) model proposed in this paper mainly includes three parts: firstly, the first part is the part of student user cognitive modeling based on TDINA model, which is described in the algorithm design of TDINA model. This part mainly analyzes and diagnoses the students' personalized cognitive ability in detail and finally obtains the prior condition that the student-knowledge point mastery matrix is used as the decomposition part of the joint probability matrix of CUPMF model recommendation algorithm. Then, the second part is the convolution neural network module of CUPMF model. This part is mainly designed for the current teaching resource recommendation algorithm not fully mining the effective implicit feature information in the resources. Its main purpose is to deeply mine the teaching resources such as test questions in different dimensions through convolution neural network and, at the same time, seamlessly integrate them into the joint probability matrix decomposition through the nonlinear transformation of the output layer. The last part is the joint probability matrix decomposition part. In this part, the probability matrix is decomposed by combining students' cognitive diagnosis information, teaching resources information, and students' score performance information on teaching resources. By using random gradient descent method, the implicit feature matrix of test questions, implicit feature matrix of students, and feature matrix of knowledge points with CNN parameters are solved, and then the possible performance of students in a certain teaching resource is predicted by these matrices, and the teaching resources whose difficulty is suitable for current student users are recommended according to their cognitive diagnosis results.

The CUPMF recommendation algorithm framework is firstly based on the information of student users' answers. Screening out the information about test questions from the test questions bank, the text information of the test questions is segmented to form a test question word set. Then, words are converted into word vectors by word embedding technology as the input of convolution neural network, and the implicit matrix *D* of test questions with CNN parameters is obtained through convolution layer, pooling layer, and output layer of nonlinear transformation of convolution neural network. The implicit matrix *D* of the test questions is taken as the implicit matrix parameter in the joint probability matrix decomposition model. Finally, combining the student-knowledge point mastery matrix obtained by TDINA model, the test question-knowledge point association matrix is marked by domain experts and the student-test question score matrix is calculated according to students' historical answer data. The implicit characteristic matrices are obtained by random gradient descent algorithm; from these implicit feature matrices, the student-test score matrix is obtained. Then, the performance of students in test teaching resources is predicted by dot product operation of implicit matrix. Finally, according to the cognitive ability of students, the recommended teaching video resources or exercise resources with appropriate difficulty are selected.

The article "Research on Teaching Resource Recommendation Algorithm Based on Deep Learning and Cognitive Diagnosis" was published in 2022. Journal: J Healthc Eng.

### 3.2. Convolution Neural Network

With the continuous development of deep learning technology, convolution neural network has been widely used by researchers, and its effect has been well verified in many network models [11–13]. Convolution neural network (CNN) can not only deeply mine the data information of various modes such as video text from different dimensions, but also strengthen the machine learning system through parameter sharing, sparse weight, and translation [14]. Among them, sparse weight means that the dimension size of convolution kernel will be far smaller than the dimension size of input data, so that convolution network can use less calculations and store fewer parameters, thus achieving efficient performance. Parameter sharing means that CNN assumes that the data have local structural characteristics, so it only needs to use different parameters in a small range of neurons, while a large range of neurons can share parameters [15]. Finally, translation invariance is based on parameter sharing, which can be intuitively understood as if the object in the input is moved, the representation in the output will be moved by the same amount. Based on the above characteristics of convolution neural network, this paper chooses CNN to mine teaching resources data. CNN framework is mainly responsible for mining potential features of teaching resources of test questions, generating implicit feature vectors of test questions and constructing implicit feature matrix representation of test questions with CNN weight parameters, which can be used for training and solving in joint probability matrix decomposition model. The convolution network framework of CUPMF model is shown in Figure 3.

The article "Research on Teaching Resource Recommendation Algorithm Based on Deep Learning and Cognitive Diagnosis" was published in 2022. Journal: J Healthc Eng.

The three categories of test questions are the content of the test questions, the options and the answers. These three parts are the complete form of the final test questions. By dividing the test questions into three categories, the neural network training is carried out separately, and the joint probability matrix decomposition model of the test questions is finally achieved.

The convolution network framework of CUPMF model consists of the following four layers.

#### 3.2.1. Word Embedding Layer

The word embedding layer converts the original test information into a dense number matrix as the input of the next convolution layer. Specifically, the test information mainly includes three parts: question stem, answer, and analysis of test questions. The three parts are segmented by word segmentation technology, and each word is converted into a word vector by randomly initializing values or pretraining word embedding model. Finally, the test questions are expressed as a dense number matrix *T*_*j*_ *∈* *R*^*P×l*^ by connecting the word vectors in the test questions information, as shown in (7), where P is the dimension of the vector and *L* is the number of word vectors.

(7) $$\begin{array}{c} T_{j}=\left[\begin{array}{ccccc} \cdots & \omega_{i-1} & \omega_{i} & \omega_{i+1} & \cdots \end{array}\right]. \end{array}$$

#### 3.2.2. Convolution Layer

Convolution layer is mainly used to extract the feature information of test questions. The essence of the feature information of test questions is different from the context information of pictures, audio or video, so it is necessary to modify the convolution network to be suitable [16]. The contextual feature *c*_*i*_^*j*^*∈ R* of a test question is extracted by the *j*-th shared weight *w*_*c*_^*j*^*∈R*^*P×w*^, and its window size *w* represents the number of surrounding words, which satisfies

(8) $$\begin{array}{c} \begin{array}{c} c_{i}^{j}=\text{fun}\left(W_{c}^{j}⊗D\left(i\times \left(i+w-1\right)\right)+b_{c}^{j}\right) \end{array}, \end{array}$$

where “ ⊗“ means convolution operation, *b*_*c*_^*j*^ ∈R is *w*_*c*_^*j*^, *R* is the deviation corresponding to *W*_*c*_^*j*^, and fun is a nonlinear excitation function (such as sigmoid, tanh, and modified linear element (ReLU)). Considering that the gradient disappears in the process of gradient descent operation, the optimization convergence process of the model becomes slow, and even the program is uncontrollable. In addition, the model may stop when the training reaches the local minimum and cannot continue to optimize. Therefore, this paper uses ReLU to avoid the gradient disappearance problem. Then, a contextual eigenvector *c*_*j*_ ∈ R^*l*-w+1^ with a weight *w*_*c*_^*j*^ is constructed by formula (8) as shown in

(9) $$\begin{array}{c} \begin{array}{c} c^{j}=\left[c_{1}^{j},c_{2}^{j},\ldots ,c_{i}^{j},\ldots ,c_{l-w^{2}+1}^{j}\right] \end{array}. \end{array}$$

Considering the limited feature information captured by using only a single shared weight, in order to output more types of feature vectors, multiple groups of shared weights are adopted in convolution layer to obtain multiple groups of feature vectors describing the feature information of test questions.

The article "Research on Teaching Resource Recommendation Algorithm Based on Deep Learning and Cognitive Diagnosis" was published in 2022. Journal: J Healthc Eng.

#### 3.2.3. Pooling Layer

After the convolution operation of the matrix composed of the test item vectors, the test item information is expressed as the characteristic moment of *n*_*c*_ horizontal dimension. The dimension of the eigenvector of test questions in matrix is not uniform; that is, the number of matrix columns is not uniform. The representation of Eigen matrix not only leads to the high dimension of vector, but also makes it difficult to construct the subsequent layer because of the disunity of each vector dimension. Therefore, this model extracts representative features from each test feature vector through pooling layer and reduces the representation of test document to *n*_*c*_ fixed-length feature vectors by constructing merging operation of fixed-length feature vectors, as shown in

(10) $$\begin{array}{c} \begin{array}{c} d_{f}=\left[\max\left(c^{1}\right),\max\left(c^{2}\right),\ldots ,\max\left(c^{j}\right),\ldots ,\max\left(c^{n_{c}}\right)\right] \end{array}. \end{array}$$

#### 3.2.4. Output Layer

The output layer is mainly responsible for nonlinear mapping of the output of the previous layer. Therefore, it is necessary to map *d*_*f*_ on the k-dimensional space of the joint probability matrix decomposition model to complete the recommendation task; that is, to generate the potential matrix of test questions by using conventional nonlinear mapping, as shown in (11):

(11) $$\begin{array}{c} \begin{array}{c} D_{j}=\tanh\left(W_{f_{2}}\left\{\tanh\left(W_{f_{1}}d_{f}+b_{f_{2}}\right)\right\}+b_{f_{2}}\right) \end{array}, \end{array}$$

wherein *W*_*f1*_*∈R*^*f×ne*^ and *W*_*f2*_*∈ R*^*k×f*^ are mapping matrices and *b*_*f1*_ and *b*_*f2*_ are deviation vectors of *W*_*f1*_, *W*_*f2*_ and *D*_*j*_ *∈* *R*_*k*_.

Finally, through the convolution and nonlinear transformation of the above hidden layers, the convolution part of CUPMF model is approximately a nonlinear function, which takes the test inscription vector as the input and outputs the implicit feature vector corresponding to each test question, as shown in

(12) $$\begin{array}{c} \begin{array}{c} D_{j}=\text{Cnn}\left(W,T_{j}\right) \end{array}, \end{array}$$

where W denotes weight and bias variables, *T*_*j*_ denotes the word vector of test *j* after sneaking through words, and *D*_*j*_ denotes the implicit feature vector of test *j*.

The article "Research on Teaching Resource Recommendation Algorithm Based on Deep Learning and Cognitive Diagnosis" was published in 2022. Journal: J Healthc Eng.

### 3.3. Joint Probability Matrix Decomposition

Matrix factorization is the most widely used model-based collaborative filtering recommendation algorithm, especially the probabilistic matrix factorization (PMF) model. Its main idea is to use matrix decomposition technology to extract low-dimensional implicit features of users and projects to predict users' interest in projects and make corresponding recommendations. Then in the field of teaching resources recommendation, it is specifically applied to knowledge point recommendation, similar resource recommendation, etc. [17]. Firstly, the student-test score matrix is decomposed by matrix decomposition technology, the implicit feature matrix of student users and test questions resources is decomposed. Then, the estimated score matrix is expressed by implicit feature matrix and fitted continuously by optimization function. Finally, the performance of students in teaching resources is predicted, and a personalized teaching resource recommendation list is generated to recommend teaching resources for students and realize teaching resource recommendation. Joint probability matrix decomposition is an association matrix organized by more user information; they are decomposed by probability matrix one by one. Compared with probability matrix decomposition, it considers more user information, and the simulated implicit features can better reflect the real situation. At the same time, it has good extensibility like probability matrix decomposition model. Therefore, this paper combines convolution neural network with joint probability matrix factorization model and proposes convolution joint probability matrix factorization (CUPMF) model, as shown in Figure 4.

The main idea of joint probability matrix decomposition of CUPMF model is that through matrix decomposition technology, the student-test score information matrix collected by the platform, the student-knowledge point mastery matrix constructed by TDINA model, and the test question-knowledge point relationship matrix manually recorded by domain experts are decomposed. The implicit feature matrix of students, knowledge points, and test questions are decomposed. The implicit feature matrix of the test questions fuses the weight parameters of convolution neural network, the original correlation information matrix is expressed by Bayesian criterion, and the real correlation information matrix data are fitted through continuous training, so as to obtain the related parameters of each implicit feature matrix. Finally, the trained implicit feature matrix predicts the students' performance in teaching resources and recommends it according to the students' mastery of knowledge points.

The article "Research on Teaching Resource Recommendation Algorithm Based on Deep Learning and Cognitive Diagnosis" was published in 2022. Journal: J Healthc Eng.

The prior probability of initialization matrix U obeys the Gaussian distribution of mean value 0 and variance *σ*_*U*_^2^ as shown in (13), and the prior probability of matrix K obeys the Gaussian distribution of mean value 0 and variance *σ*_*K*_^2^ as shown in (14). The initialization of matrix *D* is different from the traditional joint probability matrix factorization, which is mainly determined by three variables:

1. Weight W between neurons in convolution network, and the probability distribution of weight W is as (15);
2. A word vector *T*_*j*_ representing the test question *j* generated by the word embedding technique;
3. Gaussian noise *ε* ~ *N*(0, *σ*_*D*_^2^) variable.

Therefore, the implicit feature vector *D*_*j*_ generated by the CNN network of the test question *j* is represented by (16), and the probability distribution of the matrix *d* is obtained by the above equation as (17).

(13) $$\begin{array}{c} \begin{array}{c} p\left(U|\sigma_{U}^{2}\right)=\prod_{i=1}^{m}G\left(U_{i}|0,\sigma_{U}^{2}I\right) \end{array}. \end{array}$$

(14) $$\begin{array}{c} \begin{array}{c} p\left(K|\sigma_{K}^{2}\right)=\prod_{i=1}G\left(K_{i}|0,\sigma_{K}^{2}I\right) \end{array}. \end{array}$$

(15) $$\begin{array}{c} \begin{array}{c} p\left(W|\sigma_{w}^{2}\right)=\prod_{k}G\left(W_{k}|0,\sigma_{W}^{2}\right) \end{array}. \end{array}$$

(16) $$\begin{array}{c} \begin{array}{c} D_{j}=\text{Cnn}\left(W,T_{j}\right)+\varepsilon_{j} \end{array}. \end{array}$$

(17) $$\begin{array}{c} \begin{array}{c} p\left(D|W,T,\sigma_{U}^{2}\right)=\prod_{j=1}^{n}G\left(D_{j}|\text{Cnn}\left(W,T_{j}\right),\sigma_{D}^{2}I\right) \end{array}. \end{array}$$

Using the implicit vector *u*_*i*_ of student *I*, with the implicit vector *D*_*j*_ *=* *Cnn*(*w,T*_*j*_) of test *j*, it can be obtained that the score *r*_*ij*_ and probability of student *i* on test *j* obey Gaussian distribution with mean *h*(*U*_*i*_^*T*^ Cnn(*W*,*T*_*i*_)) and variance *σ*_*R*_^2^, respectively, and the mathematical expression of conditional probability distribution is as in (18). Among them, *I*_*ij*_^*R*^ is an indicator function. If student *I* has done test *j*, *I*_*ij*_^*R*^  = 1; otherwise, *I*_*ij*_^*R*^  = 0. *H*(*x*) is the sigmoid function, which maps the value of  *U*_*i*_^*T*^ Cnn(*w*,*T*_*j*_) to the (0, 1) range.

(18) $$\begin{array}{c} \begin{array}{c} p\left(R|U,D,\sigma_{R}^{2}\right)=\prod_{i=1}^{m}\prod_{j=1}^{n}{\left[G\left(r_{i,j}|h\left(U_{i}^{T}\text{Cnn}\left(W,T_{j}\right)\right),\delta_{R}^{2}I\right)\right]}^{t_{\text{ij}}^{R}} \end{array}. \end{array}$$

By the same token, from the implicit feature vector *D*_*i*_ of student *i* and the implicit feature vector *K*_*j*_ of knowledge point *j*, it can be obtained that the degree of mastery of knowledge point *j* by student *i*, *q*_*ij*_, satisfies the Gaussian distribution with mean *h*(*U*_*i*_^*T*^*K*_*j*_) and variance *σ*_*A*_^2^ and is independent, and its mathematical expression of conditional probability distribution is shown in (19), where *I*_*ij*_^*A*^ is an indicator function. If student I has mastered knowledge point *j*, *I*_*ij*_^*A*^  = 1; otherwise, *I*_*ij*_^*A*^  = 0.

(19) $$\begin{array}{c} \begin{array}{c} p\left(A|U,K,\sigma_{A}^{2}\right)=\prod_{i=1}^{m}\prod_{j=1}^{n}{\left[G\left(\alpha_{i,j}|h\left(U_{i}^{T}K_{j}\right),\delta_{A}^{2}I\right)\right]}^{I_{\text{ij}}^{A}} \end{array}. \end{array}$$

By the same token, the implicit feature vector *D*_*i*_, of test question *i*, and the implicit eigenvector *Kj* of knowledge point *j*, it can be obtained that the correlation between test question *i* and knowledge point *j* is *q*_*ij*_, which satisfies the Gaussian distribution with mean *h*(*Cnn*(*W*, *T*_*i*_)^*T*^*K*_*j*_) and variance *σ*_*Q*_^2^ and is independent, and its conditional probability distribution is shown in (20), where *I*_*ij*_^*Q*^ is the indicator function, if the knowledge point *j* is examined in the test question *i*, then *I*_*ij*_^*A*^  = 1; otherwise, *I*_*ij*_^*A*^=0.

(20) $$\begin{array}{c} \begin{array}{c} p\left(Q|D,K,\sigma_{Q}^{2}\right)=\prod_{i=1}^{m}\prod_{j=1}^{n}{\left[G\left(\alpha_{i,j}|h\left(\text{Cnn}{\left(W,T_{j}\right)}^{T}K_{j}\right),\delta_{Q}^{2}I\right)\right]}^{l_{\text{ij}}^{Q}} \end{array}. \end{array}$$

The posterior probability distributions of matrices *U*, *D*, *W,* and *K* can be obtained by Bayesian criterion.

The article "Research on Teaching Resource Recommendation Algorithm Based on Deep Learning and Cognitive Diagnosis" was published in 2022. Journal: J Healthc Eng.

The optimal solution can be solved by random gradient descent method; then, the implicit feature matrix of users, the implicit feature matrix of test questions, and the implicit feature matrix of knowledge points are calculated. Then, by multiplying the implicit feature matrix of users and the implicit feature matrix of test questions, the scores of students on test questions are predicted. Finally, according to the scores and the mastery of users' knowledge points, teaching resources with appropriate difficulty coefficients can be recommended for students.

## 4. Experiment and Evaluation

### 4.1. Data Set

In this paper, 364317 answer data were collected, named DATA0 data set. After sorting out, it was statistically determined that there were 67 knowledge points, 326 student users, and 5683 teaching resources. In addition, this paper also uses the public data sets provided by Wu et al., including FrcSub data sets and Math1 and Math2 data sets. For uniform naming, name Math1 data set DATA1 data set, Math2 data set DATA2 data set, and FrcSub data set DATA3 data set. Data sets DATA1 and DATA2 are the data of mathematics joint examination at the end of a senior high school, which are composed of students' test score data and test-knowledge point association matrix data. DATA3 data set mainly involves the subtraction of primary school scores, mainly including student-test score data and test-knowledge point related data. The score data of student users' test questions include the score data of 536 student users on 20 test questions. Among them, 0/1 scoring method is used to represent data, 1 indicates correct answer to test questions, 0 indicates incorrect answer to test questions, and the correlation matrix between test questions and knowledge points includes the correlation between 20 test questions and 8 knowledge points, and 0/1 is also used to represent the correlation relationship. If knowledge points are examined, the test questions are represented by 1, and if they are not examined, they are represented by 0. The descriptive statistics of each data set are shown in Table 1.

### 4.2. Evaluation Index

In this paper, the data are divided into training data set and test data set according to a certain proportion and randomly assigned data; that is, each data sample has the same probability as training data or test data. In this paper, the parameters of personalized recommendation method based on CUPMF model are trained by training data sets, and the recommendation effect of the algorithm is evaluated by testing data sets. In terms of evaluation indicators, this paper adopts the commonly used indicators in the recommendation system, including Precision, Recall, and F1 indicators, to evaluate the recommendation effect of teaching resources recommendation algorithm based on CUPMF model in teaching resources recommendation. Among them, F1 value combines Precision and Recall. The higher the F1 value, the higher the accuracy of the recommendation algorithm. The mathematical expressions for the specific accuracy rate, recall rate, and F1 value are defined as shown in (21).

(21) $$\begin{array}{c} \begin{array}{c} F1=\frac{2\times \text{Precision}\times \text{Recall}}{\text{Precision}+\text{Recall}} \end{array}. \end{array}$$

(22) $$\begin{array}{c} \text{Precision}=\frac{R\times Y}{R},\text{Recall}=\frac{R\times Y}{Y}. \end{array}$$

Among them, Precision represents the proportion of resources that are really suitable for student users in the recommended teaching resources, and Recall represents the proportion of all resources in the test data set that are suitable for student users in the recommended teaching resources. *Y* denotes the set of test questions that students can correctly answer in all the associated teaching resources under the knowledge set, and *R* denotes the result set of recommended teaching resources.

The article "Research on Teaching Resource Recommendation Algorithm Based on Deep Learning and Cognitive Diagnosis" was published in 2022. Journal: J Healthc Eng.

### 4.3. Analysis of Experimental Results

In order to verify the effect of the recommendation algorithm based on CUPMF model proposed in this chapter on teaching resource recommendation, in this paper, the CUPMF model recommendation algorithm is compared with some classical teaching resources recommendation methods. It includes user-based collaborative filtering (CF) recommendation method, cognitive diagnosis deterministic input noise and gate model (DITA) recommendation method, probability matrix decomposition combined with cognitive diagnosis (PMF-CD) teaching resource recommendation method, and joint probability matrix combined with cognitive diagnosis (QueRec) recommendation method.

1. User-Based collaborative filtering (CF) recommendation method: the main implementation method is to calculate the similarity among users by analyzing the historical answer data of all student users, then predict the performance of target students according to the performance of similar student users on a certain resource, and finally make recommendations according to the predicted scores combined with the difficulty of resources selected by users.
2. The recommendation method based on deterministic input noise and gate model (DINA) of cognitive diagnosis is mainly realized by using the cognitive diagnosis DNA model of educational psychology to diagnose the initial cognitive ability level of students and then select appropriate teaching resources to recommend according to the diagnosed cognitive ability level of students.
3. Combined with the probabilistic matrix decomposition (PMF-CD) teaching resource recommendation method of cognitive diagnosis: the main implementation method is to combine cognitive diagnosis model. According to the existing historical answer situation of students and the relationship between knowledge points of test questions, the students' mastery level of test questions is modeled, and then the students' mastery level of test questions is used to predict the students' answer situation by probability matrix decomposition. Finally, the corresponding teaching resources are recommended to students according to the score prediction and the difficulty of answering questions.
4. Joint Probability Matrix Decomposition (QueRec) recommendation method combined with cognitive diagnosis: its main idea is to obtain student-knowledge point mastery information through cognitive diagnosis of students, then carry out joint probability matrix decomposition according to implicit feature information of students, test questions and knowledge points, and finally recommend teaching resources according to difficulty range.

The article "Research on Teaching Resource Recommendation Algorithm Based on Deep Learning and Cognitive Diagnosis" was published in 2022. Journal: J Healthc Eng.

In the experiment, in order to observe the effect of different data sparsity on each recommendation algorithm, 70%, 50%, 30%, and 10% of all data sets are selected as test data sets, and the rest are used as training data sets. That is, when 70% of the data are randomly selected as test data, it means that the remaining 30% is used as training set to predict the test set data, and 50%, 30%, and 10% are the same. In addition, this paper divides teaching resources into simple teaching resources and complex teaching resources with the difficulty value of 0.6 as the boundary. A comparative experiment is carried out on the recommendation effect of teaching resources with different difficulties, in which the difficulty of test questions resources can be obtained by the statistics of students' historical answer data counted by multiple tests, and the rest video teaching resources and text teaching resources are manually marked by domain experts or teachers who generate and change resources.

In the CUPMF model, by adjusting the value of parameter *q*, the influence degree of data information in the question-knowledge point association matrix on the model recommendation effect can be controlled. Similarly, by controlling the value of parameter *y*, the influence degree of student-knowledge point mastery matrix on the model recommendation effect can be adjusted. In the extreme case, pa and *p* are set to 0 at the same time, which means that the influence of the corresponding two incidence matrices on the model effect is ignored, and only the influence of the student-test score matrix on the model is considered. The influence of parameters *φ*_*A*_ and *φ*_*Q*_ on the model recommendation effect (F1 value) is shown in Figures 5to 8.

From Figures 5to 8, the following conclusions can be drawn: regardless of the proportion of test data sets and whether the teaching resources are simple or complex, with the gradual increase of parameters *φ*_*A*_ and *φ*_*Q*_, the F1 value of CUPMF model recommendation algorithm increases first and then decreases slowly. Specifically, when *φ*_*A*_  = 0.5 and *φ*_*Q*_  = 1, the F1 value reaches a peak. However, when *φ*_*A*_ >0.5 or *φ*_*Q*_ > 1, the value of F1 decreases gradually; that is, the recommendation effect of CUPMF model begins to decrease gradually. The reason is that when the parameters *φ*_*A*_ and *φ*_*Q*_ are too large, the model will be more inclined to fit the training data of student-knowledge point mastery matrix and test question-knowledge point association matrix in the training process; that is, the model has overfitted the training data, which leads to the decline of recommendation accuracy. Therefore, in the CUPMF model, *φ*_*U*_,  *φ*_*B*_,  *φ*_*B*_, and *φ*_*W*_ are set to 0.001, and *φ*_*A*_ is set to 0.5. When *φ*_*Q*_ is set to 1 and the potential feature vector dimension *p* is set to 10, the recommendation effect is best.

The article "Research on Teaching Resource Recommendation Algorithm Based on Deep Learning and Cognitive Diagnosis" was published in 2022. Journal: J Healthc Eng.

In the experiment, three groups of simple teaching resources and three groups of complex teaching resources are recommended to students, and the CUPMF model method is compared with the other three methods. Experiments are carried out on the above algorithms using training sets with different sparsity degrees, and the experimental results are shown in Table 2 and Table 3.

It can be seen from Tables 2 and 3 that with the decreasing proportion of test sets, that is, the increasing proportion of training sets, the recommendation accuracy of CUPMF model in simple teaching resources and complex teaching resources is better than the other four algorithms as a whole. Specifically, when recommending simple teaching resources, the F1 value is increased by 11.61% on average compared with the other four algorithms and 1.975% on average compared with QueRec algorithm. When recommending complex teaching resources, the F1 value is increased by 11.52% on average compared with the other four algorithms and 1.875% on average compared with QueRec algorithm as a whole. The above data show that CUPMF method can effectively improve the recommendation accuracy and improve the recommendation effect. Investigating its reason, there are two main factors; on the one hand, the CUPMF model combines the TDINA model proposed in chapter three, which models the personalized cognitive diagnosis for students and generates a student-knowledge point mastery matrix with higher diagnosis accuracy, which is used as a prior condition for the joint probability matrix decomposition of CUPMF model, so that CUPMF model can fully mine the information of students' personalized cognitive ability. On the other hand, CUPMF model combines deep learning technology on the basis of joint probability model; that is, convolution neural network is seamlessly integrated into joint probability matrix decomposition model, and the hidden feature information of existing test questions resources is fully mined, so that higher recommendation accuracy can still be obtained even when student user data are sparse. From Tables 2 and 3, the algorithm is tested from the F1 values of 10%, 30%, 50%, and 70%, respectively. By comparing the test sets of different proportions, it is found that the method used in the article can reflect better performance. In Tables 2 and 3, the prediction results of teaching resources can reflect better results, indicating that the algorithm has better performance.

The article "Research on Teaching Resource Recommendation Algorithm Based on Deep Learning and Cognitive Diagnosis" was published in 2022. Journal: J Healthc Eng.

## 5. Conclusion

This paper introduces the related background of current teaching resource recommendation and then analyzes the problems in the existing teaching resource recommendation, such as insufficient consideration of students' personality, insufficient in-depth mining of teaching resource information, and insufficient recommendation accuracy. In view of the above problems, this paper proposes a teaching resource recommendation algorithm based on CUPMF model, which not only combines the student-knowledge point mastery matrix obtained by TDINA model but also integrates convolution neural network technology into the joint probability matrix decomposition model to deeply mine the information of test questions resources. Then, according to students' cognitive ability level and their individual needs, a resource recommendation list is generated, and teaching resources with appropriate difficulty are recommended for them. Finally, experimental analysis is carried out on Guangdong Education Cloud Platform and other three public real data sets, and the results show that the recommendation effect of this algorithm is better than the three existing recommendation algorithms as a whole in F1 index. It is proved that the recommendation method based on CUPMF model can effectively improve the recommendation effect and accuracy.

## Figures and Tables

**Figure 1:** Flow chart of cognitive diagnosis algorithm of TDINA model.

**Figure 2:** Schematic diagram of R matrix and Q matrix.

**Figure 3:** Framework diagram of convolution network of CUPMF model.

**Figure 4:** Frame diagram of joint probability matrix decomposition of CUPMF model.

**Figure 5:** Influence of parameter *φ*_*A*_ on F1 value when recommending simple teaching resources.

**Figure 6:** Influence of parameter *φ*_*A*_ on F1 value when recommending complex teaching resources.

**Figure 7:** Influence of parameter *φ*_*Q*_ on F1 value when recommending simple teaching resources.

**Figure 8:** Influence of parameter *φ*_*Q*_ on F1 value when recommending complex teaching resources.

**Table 1:** Data set statistics table.

Data set	Number of students	Number of teaching resources	Knowledge points
DATA0	326	5683	67
DATA1	4209	20	11
DATA2	3911	20	16
DATA3	536	20	8

The article "Research on Teaching Resource Recommendation Algorithm Based on Deep Learning and Cognitive Diagnosis" was published in 2022. Journal: J Healthc Eng.

**Table 2:** F1 value table of prediction results of simple teaching resources.

Recommendation algorithm	Test set ratio			
	70%	50%	30%	10%
User-based CF	0.501	0.506	0.532	0.479
DINA	0.539	0.606	0.617	0.699
PMF-CD	0.695	0.632	0.639	0.701
QueRec	0.690	0.701	0.737	0.768
CUPMF	0.722	0.753	0.781	0.719

**Table 3:** F1 value table of prediction results of complex teaching resources.

Recommendation algorithm	Test set ratio			
	70%	50%	30%	10%
User-based CF	0.483	0.615	0.593	0.606
DINA	0.693	0.653	0.706	0.741
PMF-CD	0.687	0.715	0.721	0.774
QueRec	0.759	0.789	0.797	0.832
CUPMF	0.791	0.787	0.823	0.851

## Data Availability

The experimental data used to support the findings of this study are available from the corresponding author upon request.
